# Comparative Study on Diagnosis Value of Contrast-Enhanced Ultrasound and Contrast-Enhanced Computed Tomography after Treating Advanced Renal Cancer Patients with Yiqi Jiedu Decoction

**DOI:** 10.1155/2021/5763618

**Published:** 2021-10-26

**Authors:** Yupeng Lan, Tengfen Gong, Ruhai Zhou, Meng Wu, Zhenzhen Liu

**Affiliations:** ^1^Department of Ultrasound, The Affiliated People's Hospital of Ningbo University, Ningbo 315040, Zhejiang, China; ^2^Department of Traditional Chinese Medicine, The Affiliated People's Hospital of Ningbo University, Ningbo 315040, Zhejiang, China; ^3^Department of Ultrasound Medicine, Peking Union Medical College Hospital, Beijing 100032, China

## Abstract

**Objective:**

To compare and analyze the diagnosis value of contrast-enhanced ultrasound (CEUS) and contrast-enhanced computed tomography (CECT) after treating advanced renal cancer patients with Yiqi Jiedu decoction.

**Methods:**

The case data of 60 patients diagnosed with advanced renal cancer from January 2013 to January 2021 at the Affiliated People's Hospital of Ningbo University were retrospectively analyzed, 30 patients who accepted the conventional treatment were included in the control group, and the rest treated with Yiqi Jiedu decoction on the basis of conventional treatment were included in the study group. After treatment, patients in both groups received the CEUS and CECT examinations, the diagnosis efficacy of both examinations was evaluated with the ROC curve, and the overall survival (OS) of patients was analyzed.

**Results:**

No significant between-group differences in the general information were observed (*P* > 0.05); the clinical remission rate and disease control rate were not significantly different between the two groups (*P* > 0.05); the enhancement and attenuation, degree of enhancement, uniformity of enhancement, and pseudocapsule sign of the CEUS and CECT examinations were not remarkably different (*P* > 0.05); according to the results of CEUS and CECT examinations, the maximum diameters of tumor after treatment were smaller in the study group than in the control group, but with no significant between-group difference (*P* > 0.05); in addition, there were no obvious differences in determining the maximum diameter of tumor by CEUS and CECT (*P* > 0.05), and the results of the maximum diameter of tumor determined by CEUS, CECT, and pathological specimen were not statistically different (*P* > 0.05); as for the diagnosis efficacy, the result was CEUS + CECT > CEUS > CECT; and the OS of patients in the study group was longer than those in the control group.

**Conclusion:**

The patients treated with Yiqi Jiedu decoction obtain longer OS, and the application value of CEUS combined with CECT in the treatment effect and prognosis of patients with advanced renal cancer is higher.

## 1. Introduction

The incidence of kidney cancer in urinary tract tumors in China is second only to that of bladder tumors, which accounts for 3-4% of malignant tumors in adults and is increasing year by year. Currently, the clinical diagnosis of renal cancer mainly relies on imaging examination because there is no generally accepted tumor marker available. Contrast-enhanced ultrasound (CEUS) and contrast-enhanced computed tomography (CECT) are emerging technologies in ultrasound diagnostics in recent years, which can reflect the blood perfusion characteristics of pathological tissue and have high diagnostic values in the early renal cancer, progressive renal cancer, and recurrent renal cancer [1–4]. Yiqi Jiedu decoction has the efficacy of invigorating qi, promoting diuresism, and removing toxicity, and it has been applied clinically as an adjuvant regimen of traditional Chinese medicine for renal cancer patients in our hospital for many years, achieving better clinical outcomes [5]. Some studies found that both CEUS and CECT can effectively evaluate cancer patients' treatment performance by determining the intratumoral blood perfusion parameters before and after treatment, which can be used to guide subsequent treatment options [6–8]. Based on this, CEUS and CECT examinations were carried out for 60 patients with advanced renal cancer treated in our hospital, and the diagnostic value of both after treating such patients with Yiqi Jiedu decoction was further evaluated in this study.

## 2. Data and Methods

### 2.1. Inclusion Criteria

(1) The patients had parenchymatous space-occupying lesion in the kidney; (2) the patients' estimated survival was more than 6 months; (3) the clinical data of patients were complete; (4) the patients and their family members agreed to join the study and signed the informed consent; (5) the lesion was on the one side; and (6) the patients met the TCM treatment indications of Yiqi Jiedu decoction.

### 2.2. Exclusion Criteria

(1) The patients had simple cyst of the kidney; (2) the patients had other severe organic diseases or coagulation disorder; (3) the patients suffered from other malignant tumors; (4) the follow-up time was less than 1 month; (5) pregnant or lactating women; (6) the patients presented communication disorders or cognitive disorders; and (7) the patients had contraindication of CEUS and CECT examinations.

### 2.3. Grouping

The case data of 60 patients diagnosed with advanced renal cancer at the Affiliated People's Hospital of Ningbo University from January 2013 to January 2021 were retrospectively analyzed, 30 patients who accepted the conventional treatment were included in the control group, and the rest treated with Yiqi Jiedu decoction on the basis of conventional treatment were included in the study group. The implementation of the study was monitored by the Ethics Committee of the Affiliated People's Hospital of Ningbo University.

### 2.4. Methods

All patients received the conventional chemoradiotherapy according to their condition, and on this basis, those in the study group took one dose of Yiqi Jiedu decoction (20 g of Mongolian milkvetch root, 20 g of Largehead Atractylodes Rhizome, 30 g of Solomonseal Rhizome, 15 g of tuber of multiflower knotweed, 30 g of *Hedyotis*, 15 g of Barbated Skullcup herb, 15 g of Giant Knotweed Rhizome, 15 g of *Isatis* root, and 15 g of Danshen root) daily in two split times (in the morning and the evening) for 60 days [9, 10]. After that, all patients received the CEUS and CECT examinations.

#### 2.4.1. CEUS Test

Two focus points under the lesion were set with the ultrasonography (model: Siemens Sequoia 512) and probes (model: 4C1; frequency: 2.0–4.5 MHz) under MI 0.21 [11, 12], which were applied for all patients. The freeze-dried powder of the SonoVue contrast agent was dissolved and shaken with 5 ml of normal saline into milk white liquid; then, the patients were administered with 1.2 ml of it via elbow vein bolus injection and flushed with 5 ml of normal saline (i.e., the contrast agent was completely injected within 3–5 s); meanwhile, the CPS mode and timekeeping were initiated to observe the start time of ultrasound contrast enhancement and attenuation of kidney cortex, medulla, and lesion, record the lesion form, size, blood flow, and boundary, and videotape the whole process. The TIC curve was obtained by the analysis software to analyze various parameters and compare the enhancing intensity between lesion and surrounding normal renal parenchyma to determine the enhancing intensity of ultrasound contrast. For patients with a poor imaging effect or incomplete image, a second CEUS could be carried out 10 min after the first contrast.

#### 2.4.2. CECT Test

The patients were in the spine position and scanned with the Siemens SOMATOM Sensation 64-Slice CT from their porta hepatis plane to lower pole of the kidney with routine plain scan first and then contrast-enhanced scan. During the contrast-enhanced scan, 80 ml of nonionic iodine contrast agent (specification: 300 mgI/ml) was administered via elbow vein injection with the binocular high-pressure syringe under the rate of 3-4 ml/s; then, 30 ml of normal saline was injected under the rate of 3 ml/s, and after that, the arterial phase, portal venous phase, and scanning were delayed for, respectively, 28 s, 70 s, and 180 s. The scan conditions were set as follows: gantry rotation was 0.33 s per rotation, reference current was 500 mAs, tube potential was 120 kVp, detector straight line was 32 × 0.6 mm, and thread interval was 0.65–1.3 mm; for the conventional reconstruction images, both the slice thickness and slice interval were 8 mm, and for the thin reconstruction images, 1 mm, and sagittal or coronal scanning was performed on thin slice reconstructed images with a thickness of 4–6 mm and FOV of 35–45 cm [13].

### 2.5. Observation Indexes

  General information: the patients' general information included their age, tumor diameter, gender, affected side of tumor, tumor location, clinical manifestations, and pathological type.
  Clinical efficacy: according to the Response Evaluation Criteria in Solid Tumors (RECIST) [14], the clinical efficacy was classified into complete response (CR), partial response (PR), stable disease (SD), and progressive disease (PD). The clinical remission rate = (CR + PR)/total number × 100%, and the disease control rate = (CR + PR + SD)/total number × 100%.
  Follow-up observation: the follow-up visits were conducted after the first month of treatment, mainly including imaging examination, serum tumor marker, and routine physical examinations such as the routine blood test, routine urinalysis, erythrocyte sedimentation rate (ESR), and hepatic and kidney function.

### 2.6. Statistical Processing

In this study, the between-group differences in data were calculated by SPSS22.0, the picture drawing software was GraphPad Prism 7, the enumeration data were expressed by (*n* (%)) and examined with the *X*^2^ test, the measurement data were expressed by ($\bar{x}\pm s$) and examined with the *t*-test, and differences were considered statistically significant at *P* > 0.05.

## 3. Results

### 3.1. General Information

No significant differences in the general data between the two groups were observed (*P* > 0.05), indicating no statistical significance.  Table 1 provides the specific data.

### 3.2. Clinical Efficacy of Patients in Both Groups

No statistical differences in the clinical remission rate and disease control rate of patients between the two groups were observed (*t* = 0.073, 0.082; *P*=0.787, 0.774) (Figure 1).

The control group had 2 CR cases, 8 PR cases, 12 SD cases, and 8 PD cases, and the clinical remission rate and disease control rate were 33.33% (10 cases) and 73.33% (22 cases), respectively.

The study group had 2 CR cases, 9 PR cases, 10 SD cases, and 9 PD cases, and the clinical remission rate and disease control rate were 36.67% (11 cases) and 70% (21 cases), respectively.

### 3.3. Imaging Characteristics of Patients with Advanced Renal Cancer on CEUS and CECT Scans

No significant differences in the ultrasound characteristics including enhancement and attenuation, degree of enhancement, uniformity of enhancement, and pseudocapsule sign on CEUS and CECT scans of 60 advanced renal cancer patients were observed (*P* > 0.05) (Table 2 and Figure 2).

### 3.4. Changes in the Maximum Diameters of Tumor before and after Treatment

According to the CEUS and CECT tests, the maximum diameters of tumor in patients were smaller in the study group than in the control group, but the between-group differences were not significant (*P* > 0.05); in addition, there were no obvious differences in determining the maximum diameter of tumor by CEUS and CECT (*P* > 0.05) (Table 3); the results of the maximum diameter of tumors determined by CEUS, CECT, and pathological specimen were not statistically different (*P* > 0.05) (Table 4).

### 3.5. Diagnosis Efficacy of CEUS and CECT for Advanced Renal Cell Carcinoma Patients

Taking the postoperative pathological examination as the golden standard, the diagnosis efficacy of CEUS and CECT for advanced renal cell carcinoma was evaluated with the ROC curve, and the result was CEUS + CECT > CEUS > CECT (Figure 3 and Table 5).

### 3.6. Comparison of Patients' OS between the Two Groups

The difference in the follow-up visit time (months) between the study group and the control group was not significant (13.68 ± 2.11 vs. 13.94 ± 2.30, *t* = 0.456, *P*=0.650); the patients' OS was longer in the study group than in the control group, as shown in Figure 4.

## 4. Discussion

Renal cell carcinoma has an incidence rate second only to bladder cancer among urinary tract tumors in China. According to epidemiological investigation, renal cell carcinoma accounts for approximately 2-3% of malignant tumors in adults, with an average standardized morbidity of 3.7/100,000 that is obviously increasing in recent years [15, 16]. Renal cell carcinoma has a very rapid disease progression and is the most lethal malignancy of all urinary tumors. Although surgery is the optimal treatment for renal cell carcinoma, nearly half of the patients are advanced at the time of first diagnosis and lose the opportunity of surgery, and a large number of clinical studies have shown that the disease is not sensitive to radiation therapy, so postoperative chemoradiotherapy is not a significant predictor of improved patient survival [17–20]. Therefore, Yiqi Jiedu decoction is commonly used in the clinic to assist renal cancer treatment, in the hope of enhancing drug efficacy, reducing drug toxic and side effects and tumor volume, and lowering the clinical stage, so as to enable the inoperable patients to receive surgery and even prolong their survival. To better control the condition of renal cancer patients, especially those in the advanced stage, effective diagnostic modalities must be adopted to evaluate their treatment performance, guide subsequent treatment options, and prevent remetastasis and recurrence. With the continuous development of ultrasound contrast agents and contrast imaging technology, CEUS can observe the intratumoral blood perfusion in real-time, dynamically and continuously, which makes up for the deficiency of two-dimensional ultrasound, color ultrasound, CT, and other examinations in the diagnosis of renal cell carcinoma, and provides a new method for qualitative diagnosis.

In this study, the clinical remission rate and disease control rate of patients were not significantly different between the two groups (*P* > 0.05), which was consistent with the report of Choi et al. [15]. In addition, according to the results of CEUS and CECT examinations, the maximum diameters of tumor after treatment were smaller in the study group than in the control group, but the between-group difference was not significant (*P* > 0.05), indicating that Yiqi Jiedu decoction could reduce the maximum diameter of tumor for advanced renal cell carcinoma patients, but the result was not statistically significant. The results of the maximum diameter of tumor determined by CEUS, CECT, and pathological specimen were not statistically different (*P* > 0.05); the diagnosis efficacy of CEUS and CECT on renal cell carcinoma was evaluated by the ROC curve, and the result was CEUS + CECT > CEUS > CECT, implying that the CEUS obtained a better diagnosis efficacy than CECT, both of them could be used as the imaging examination for measuring the size of renal tumor, and the correctness of their combination was higher. Also, the enhancement and attenuation, degree of enhancement, uniformity of enhancement, and pseudocapsule sign in CEUS and CECT scans for 60 patients with advanced renal cancer were not significantly different (*P* > 0.05), denoting that both CEUS and CECT could identify the renal cell carcinoma by enhancing the diffusivity and centrality.

Compared with CECT, CEUS is simple to operate, and the contrast medium used is iodine-free gas-filled microbubbles, which is noninvasive, nonallergic, nonradiating, and safer, and can be discharged all over the lung in about 10 min without liver and kidney toxicity; moreover, the ultrasound contrast agent is essentially the blood pool imaging agent that stays only intravascularly, thus accurately reflecting the characteristics of tissue microvascular perfusion; finally, CEUS is also capable of real-time, dynamic, and continuous monitoring of the phasic changes in blood perfusion in tumor lesions; in particular, its display of the microvasculature of tumors and low blood flow is better than CT [21–24]. However, for double renal lesions or multiple lesions on the one side, CEUS can only obtain contrast perfusion imaging of relatively local or adjacent lesions, and lesions in different parts are difficult to show simultaneously; for deep or superficially special tumors, multiple contrasts are necessary to achieve better results; besides, contrast agents are expensive, so it is difficult to widely promote their application. The study also has the following deficiencies. For example, it was a single center study with a small sample size, and the in-depth exploration of study dimensions with insignificant differences still requires a larger sample size. In addition, the analysis of patients' quality of prognosis survival and time to disease progression was not addressed.

In conclusion, patients treated with Yiqi Jiedu decoction obtain longer OS, the diagnostic sensitivity and accuracy of CEUS for advanced renal cancer are better than those of CECT, but the combination of CEUS and CECT is more valuable in the treatment effect and prognosis of patients with advanced renal cancer.

## Figures and Tables

**Figure 1:** Comparison of patients' clinical efficacy between the two groups (%). Note: the horizontal axis indicates the evaluation dimensions, and the vertical axis indicates the percentage (%).

**Figure 2:** CEUS and CECT scans imaging of patients with advanced renal cancer note. (a) CEUS scan for renal clear cell carcinoma with pseudocapsule sign around. (b) The image of the pseudocapsule formation in a case with renal clear cell carcinoma. (c) CEUS scan for renal cell carcinoma with no tumor enhancement. (d) CEUS scan for renal cell carcinoma showing uniform hyperenhancement of the tumor.

**Figure 3:** ROC curve.

**Figure 4:** Patients' OS of the two groups. Note: the horizontal axis indicates the survival time (month), the vertical axis indicates the survival rate (%), and ...... indicates the survival time corresponding to the median survival rate of patients in both groups.

**Table 1:** Statistics of patients' general information of the two groups (*n* = 30).

Observation indicator	Control group	Study group	*t*/*X*^2^	*P*
Age (years)	50.48 ± 8.36	51.13 ± 8.52	0.298	0.767
Tumor diameter (cm)	3.51 ± 2.23	3.47 ± 2.31	0.068	0.946
Gender (male)	11 (36.67%)	13 (43.33%)	0.278	0.596
Affected side			0.268	0.605
Left	17 (56.67%)	15 (50%)		
Right	13 (43.33%)	15 (50%)		
Tumor position				
Upper pole of the kidney	7 (23.33%)	6 (20%)	0.098	0.754
Midpole of the kidney	12 (40%)	14 (46.67%)	0.272	0.602
Lower pole of the kidney	11 (36.67%)	10 (33.33%)	0.073	0.787
Clinical manifestation				
Painless hematuria	11 (36.67%)	9 (30%)	0.300	0.584
Lumbago	4 (13.33%)	5 (16.67%)	0.131	0.718
Hematuria with lumbago	15 (50%)	16 (53.33%)	0.067	0.796
Pathological type			0.341	0.559
Locally advanced renal cell carcinoma	23 (76.67%)	21 (70%)		
Metastatic renal cell carcinoma	7 (23.33%)	9 (30%)		

**Table 2:** Imaging characteristics of patients with advanced renal cancer on CEUS and CECT scans (*n* (%)).

Characteristic dimension	CEUS	CECT	*X* ^2^	*P*
Enhancement and attenuation			1.905	0.168
Fast enhancement and fast attenuation	7 (11.67)	10 (16.67)		
Fast enhancement and slow attenuation	39 (65)	38 (63.33)		
Slow enhancement and fast attenuation	4 (6.67)	7 (11.67)		
Slow enhancement and slow attenuation	10 (16.67)	5 (8.33)		
Degree of enhancement			0.745	0.388
High	44 (73.33)	45 (75)		
Low	16 (26.67)	12 (20)		
None	0 (0)	3 (5)		
Uniformity of enhancement			0.534	0.465
Yes	27 (45)	31 (51.67)		
No	33 (55)	29 (78.33)		
Pseudocapsule sign			0.310	0.577
Yes	26 (43.33)	23 (38.33)		
No	34 (56.67)	37 (61.67)		

**Table 3:** Changes in the maximum diameters of tumor before and after treatment (mm).

Group	CEUS		CEUS	
	Before treatment	After treatment	Before treatment	After treatment
Control group	45.66 ± 10.81	28.59 ± 7.08	46.17 ± 10.98	28.01 ± 7.05
Study group	45.16 ± 10.75	25.81 ± 6.15	46.20 ± 11.04	25.19 ± 6.27
*t*	0.180	1.624	0.011	1.637
*P*	0.858	0.110	0.992	0.107

**Table 4:** Comparison of the maximum diameters of tumor after treatment determined by CEUS, CECT, and pathological specimen (mm).

Method	Maximum diameter of tumor
CEUS	26.55 ± 6.23
CECT	26.38 ± 6.25
Pathological specimen	26.11 ± 6.19
*t*_CEUS-pathological_/*P*_CEUS-pathological_	0.274/0.785
*t*_CEUS-pathological_/*P*_CEUS-pathological_	0.168/0.867

**Table 5:** Area under the curve.

Variable of test result	Area	Standard error	Asymptotic Sig.	Asymptotic 95% CI	
				Lower limit	Upper limit
CEUS + CECT	0.983	0.019	0.100	0.000	1.000
CEUS	0.949	0.041	0.126	0.000	1.000
CECT	0.941	0.046	0.133	0.000	1.000

## Data Availability

The data used to support the findings of this study are available from the corresponding author upon request.
